The article "Cost-effectiveness of two long-lasting insecticidal nets delivery models in mass campaign in rural Mozambique" was published in 2019. Journal: BMC Res Notes.

# Cost-effectiveness of two long-lasting insecticidal nets delivery models in mass campaign in rural Mozambique

**DOI:** 10.1186/s13104-019-4620-6

**Published:** 2019-09-14

**Authors:** Jorge A. H. Arroz, Baltazar Candrinho, Chandana Mendis, Melanie Lopez, Maria do Rosário O. Martins

**Affiliations:** 1 World Vision International, Maputo, Mozambique; 2 National Malaria Control Programme, Maputo, Mozambique; 3 World Vision Inc., Federal Way, WA USA; 4 Global Health and Tropical Medicine, GHTM, Instituto de Higiene e Medicina Tropical, IHMT, Universidade Nova de Lisboa, UNL, Rua da Junqueira 100, 1349-008 Lisbon, Portugal

**Keywords:** Long-lasting insecticidal nets campaign, Universal health coverage, New and standard delivery model, Cost-effectiveness analysis, Malaria, Mozambique

## Abstract

**Objective:**

The aim is to compare the cost-effectiveness of two long-lasting insecticidal nets (LLINs) delivery models (standard vs. new) in universal coverage (UC) campaigns in rural Mozambique.

**Results:**

The total financial cost of delivering LLINs was US$ 231,237.30 and US$ 174,790.14 in the intervention (302,648 LLINs were delivered) and control districts (219,613 LLINs were delivered), respectively. The average cost-effectiveness ratio (ACER) per LLIN delivered and ACER per household (HH) achieving UC was lower in the intervention districts. The incremental cost-effectiveness ratio (ICER) per LLIN and ICER per HH reaching UC were US$ 0.68 and US$ 2.24, respectively. Both incremental net benefit (for delivered LLIN and for HHs reaching UC) were positive (intervention deemed cost-effective). Overall, the newer delivery model was the more cost-effective intervention. However, the long-term sustainability of either delivery models is far from guaranteed in Mozambique’s current economic context.

## Introduction

Using long-lasting insecticidal nets (LLINs) can reduce malaria morbidity and mortality [1–3]. Worldwide funding for malaria control fell by 8% between 2013 and 2014 [4]. Funding for the provision of LLINs can continue to decrease [5] and it is necessary to ensure cost-effective and sustainable LLINs delivery models.

Spending on malaria control commodities is estimated to have increased globally from about US$ 40 million in 2004 to about US$ 1.6 billion in 2014, where LLINs were responsible for 63% of total spending in 2014 (US$ 1 billion) [5]. Due to high burden of malaria in the sub Saharan Africa and the strategy of universal LLINs coverage, most of the international funding in 2014 was spent in the WHO African Region. In Mozambique, half of the international funding for malaria intervention went to mosquito nets [5].

Most of the economic studies do not compare the distribution of LLINs through the same mechanisms or channel. Recently, Ntuku et al. [6] evaluated a fixed delivery strategy and a door-to-door strategy. Their findings show that the fixed delivery strategy achieved a higher LLIN coverage at lower delivery cost compared with the door-to-door strategy.

The article "Cost-effectiveness of two long-lasting insecticidal nets delivery models in mass campaign in rural Mozambique" was published in 2019. Journal: BMC Res Notes.

In 2015, Mozambique piloted a new model of LLIN delivery in campaign [7]. Two rural districts were intervened with a new LLIN delivery model, and two served as the control, maintaining the standard delivery model. Results of this pilot showed that 87.8% (302,648) of planned LLINs were distributed in the intervention districts compared to 77.1% (219,613) in the control districts [7].

The objective of this research is to compare the cost-effectiveness of the two delivery models in mass campaigns in rural Mozambique, and establish the most cost-effective LLIN delivery model.

## Main text

### Methods

#### Setting and location

The study was conducted in four rural districts of Mozambique. Two districts served as intervention (with the new delivery model); and two served as control (with standard delivery model). These districts were selected based on pragmatic criteria described elsewhere [7]. All four districts are rural, with limited access to health services, and low health, social and economic indicators [7, 8].

#### Study design

An observational and cross-sectional study with cost-effectiveness analysis component was carried out using secondary data from the pilot study conducted between October and December 2015 [7].

#### Collection of cost data

The campaign costs were retrospectively collected from the providers’ perspective. The costs considered were related to training of personnel, allowances, LLINs warehouse storage, LLIN transportation vehicles rental, and materials production (pamphlets, coupons, stickers, etc.).

These costs were aggregated into four categories: (1) micro-planning; (2) LLIN storage; (3) LLIN transport; (4) mobilization and training at district level, household registration, and LLIN distribution.

Costs were collected in local currency and United States Dollars (US$). In 2015, the exchange rate was: 1 US$ = 42.00 Meticais. No adjustment for inflation was undertaken since all cost were paid in 2015. No discount rate was applied since the temporal universe of analysis did not exceed 1 year.

#### Comparators: the two delivery models

Both delivery models are community-based. One delivery model allocates LLINs based on the assumption of one LLINs for every two persons in a household (intervention districts), and another the number of LLINs is allocated based on assumptions around households members sleeping patterns (control districts). A comprehensive description of the models and pitfalls associated during implementation are reported elsewhere [7, 8].

The article "Cost-effectiveness of two long-lasting insecticidal nets delivery models in mass campaign in rural Mozambique" was published in 2019. Journal: BMC Res Notes.

#### Measurement of effectiveness

Two endpoints were used to measure the effects of the campaign in the intervention and control districts: (i) number of LLINs delivered; (ii) households (HHs) achieving universal coverage (UC) target (one LLIN for every two persons). The number of HHs achieving UC was estimated according to the following steps:

- Step 1: percentage of HHs achieving UC—[70.8% (95% CI 67.6–74.0) in the intervention districts, and 59.6% (95% CI 56.2–63.0) in the control districts] [8];
- Step 2: registered HHs multiplied the step 1 results (136,985 HHs were registered in the intervention districts, and 120,246 HHs were registered in the control districts [7]).

#### Cost-effectiveness analyses

The following cost-effectiveness measures were calculated: (i) average cost-effectiveness ratio (ACER) per LLIN delivery; (ii) ACER per HH achieving UC; (iii) incremental cost-effectiveness ratio (ICER); and (iv) incremental net benefit (INB).

- The ACER per LLIN delivered and ACER per HH achieving UC was calculated by dividing the total implementation cost by the number of LLINs delivered and number of HHs achieving UC, respectively.
- The ICER was calculated by dividing the difference between the total cost by the difference of effects in the intervention and control districts.
- The INB was calculated by valuing additional effect (∆E) in dollars and then subtracting the associated additional cost (∆C): INB = (∆E × λ) − ∆C, where λ is willingness to pay (WTP) for a 1-unit gain of effect [9].

#### Willingness to pay (WTP) and decision rule on cost-effectiveness

Three WTP was adopted:

- WTP 1) for LLINs delivered (US$ 1.32 per LLIN—adopted by the Global Fund for Mozambique in-country mass free campaign budget planning [10]);
- WTP 2) for LLINs delivered plus LLIN purchases cost (US$ 9.12 per LLIN − US$ 1.32 + US$ 7.8 which was the maximum inter-quartile purchase cost for the period 2005–2012 [11]); and
- WTP 3) for HHs achieving UC (US$ 3.30 per household). This third WTP was determined by multiplying the average number of HH members (five) [7] by US$ 1.32, and dividing by two (one LLIN for every two persons).

The cost-effectiveness decision rule was based on INB results. Two INB was calculated: INB for delivered LLIN (using WTP 1 and 2) and INB for HHs achieving UC (using WTP 3). A positive INB means that the new intervention extra benefits (∆E × λ) outweighs its extra costs (∆C), i.e., the new intervention is deemed cost-effective. Conversely, when INB is less than 0 (negative INB), the new intervention is not cost-effective [9].

The article "Cost-effectiveness of two long-lasting insecticidal nets delivery models in mass campaign in rural Mozambique" was published in 2019. Journal: BMC Res Notes.

#### Sensitivity analysis

A one-way sensitivity analysis was performed on the following parameters and assumptions: (i) free warehouses; (ii) transport cost (± 50%); and (iii) costs of LLINs purchase (− 25%, − 50%). Base case cost analysis was used to calculate the percentage of deviation. For the first two parameters, the base case was the ACER and ICER per LLIN delivered. For the third parameter, the base case was also ACER and ICER per LLIN delivered but also included the 2014 purchase cost of US$ 3.63 per LLIN for the planned 344,770 LLINs in the intervention and 284,873 LLINs in the control districts.

The US$ 3.63 per LLIN was based on the unit cost for Disease Control Technologies Royal Sentry^®^ rectangular LLINs 190 × 180 × 180 cm of US$ 3.19; procurement fee 1.50%; outbound transport charges 11.94%; transport insurance charges 0.14%; question and answer charges 0.09%; and pre-shipment inspection charges 0.12%.

### Results

#### Financial costs of the LLIN campaign

The total financial cost of the campaign from the providers’ perspective was US$ 231,237.30 and US$ 174,790.14 in the intervention and the control districts, respectively. Cost activity category 4 and 3 comprised around 43% and 38% in the intervention districts and 50% and 41% in the control districts, respectively. Cost activity category 4 were US$ 0.06/LLIN higher in the control districts. The ACER per LLIN delivered was US$ 0.76 and US$ 0.80 in the intervention and control districts, respectively—Table 1. The ACER for HHs achieving UC was lower in the intervention districts (US$ 2.38 vs. US$ 2.43)—Table 2.

**Table 1:** Total cost and cost per LLIN delivered (US$) for each category in the intervention and control districts

	Intervention (new delivery model)		Control (standard delivery model)	
LLIN delivered	302,648		219,613	

Aggregated and standardized categories	Cost	%	Cost	%
1. Micro-planning	6184.85	2.7	5580.84	3.2
ACER per LLIN delivered	0.02		0.03	
2. LLIN warehouse storage	6983.76	3.0	6880.33	3.9
ACER per LLIN delivered	0.02		0.03	
3. LLIN transport	86,908.64	37.6	71,007.48	40.6
ACER per LLIN delivered	0.29		0.32	
4. Mobilization, trainings at district level, household registration, and LLIN distribution	99,105.53	42.9	86,736.97	49.6
ACER per LLIN delivered	0.33		0.39	
4.1 Coupons and Stickers production	32,054.52	13.9	NA	NA
ACER per LLIN delivered	0.11		NA	
4.2 Household registration data analysis	NA	NA	4584.52	2.6
ACER per LLIN delivered	NA		0.02	
Total cost	231,237.30	100.0	174,790.14	100.0
ACER per LLIN delivered	0.76		0.80	

Household registration data analyses were not necessary in the intervention districts; coupons and stickers were not used in the control districts

*NA* not applicable

The article "Cost-effectiveness of two long-lasting insecticidal nets delivery models in mass campaign in rural Mozambique" was published in 2019. Journal: BMC Res Notes.

**Table 2:** Comparative cost-effectiveness results in the intervention and control districts

Effects and cost-effectiveness indicators	Intervention (new delivery model)	Control (standard delivery model)
Delivered LLINs	302,648	219,613
Registered Households	136,985	120,446
HHs achieving UC (%)	70.8	59.6
HHs with UC	96,985	71,786
Total cost (U$S)	231,237.30	174,790.14
ACER for HHs achieving UC (U$S)	2.38	2.43
∆ Cost (U$S)	56,447.16	
∆ Effect (LLINs delivered)	83,035	
∆ Effect (HHs achieving UC)	25,199	
ICER for delivered LLIN (U$S)	0.68	
ICER for HHs achieving UC (U$S)	2.24	
INB for delivered LLIN (U$S)	+ 53,159.04	
INB for HHs achieving UC (U$S)	+ 26,709.54	

#### Cost-effectiveness and decision rule

The overall ICER to deliver one additional LLIN was US$ 0.68, with a positive INB (intervention deemed cost-effective), i.e., a saving of more than US$ 50,000 per LLIN delivered would result from switching from the standard to new delivery model (with U$S 1.32 as WTP)—Table 2. The overall ICER for one households reaching universal coverage was US$ 2.24, with a positive INB, i.e., a saving of more than US$ 26,000 per household reaching universal coverage would result from switching from the standard to new delivery model (with U$S 3.30 as WTP)—Table 2.

#### Sensitivity analysis

After a sensitivity analysis, the ACER per LLIN delivered remained at a lower rate (less sensitive) in the intervention districts rather than in the control districts, i.e., the results of ACER per LLIN delivered remain robust. The cost-effectiveness of the new delivery model also remained sustained for all the parameters tested (positive INB even using WTP 2)—Table 3.

**Table 3:** Deterministic one-way sensitivity analysis of cost estimates to key assumptions

Parameter tested	Control/intervention districts	Cost (US$)	ACER_LLIN_	% ACER_LLIN_ deviation	ICER_LLIN_	% ICER_LLIN_ deviation	INB_LLIN_
Free warehouse	Control	167,909.81	0.76	− 4.43			
	Intervention	224,253.54	0.74	− 2.50	0.68	− 0.18	53,262.46
Transport cost (+ 50%)	Control	210,293.88	0.96	19.70			
	Intervention	274,691.63	0.91	19.42	0.78	14.09	45,208.45
Transport cost (− 50%)	Control	139,286.40	0.63	− 20.72			
	Intervention	187,782.98	0.62	− 18.36	0.58	− 14.08	61,109.62
LLIN purchase cost + delivery cost	Control	1,214,576.59	5.53	NA			
	Intervention	1,489,647.80	4.92	NA	3.31	NA	482,207.98
Less 25% LLIN purchase cost + delivery cost	Control	954,629.98	4.35	− 21.39			
	Intervention	1,175,045.18	3.88	− 21.09	2.65	− 19.80	536,864.00
Less 50% LLIN purchase cost + delivery cost	Control	694,683.36	3.16	− 42.80			
	Intervention	860,442.55	2.84	− 42.21	2.00	− 39.69	591,520.01

*NA* not applicable because is the new base case with the inclusion of LLIN purchase cost into delivery cost

The article "Cost-effectiveness of two long-lasting insecticidal nets delivery models in mass campaign in rural Mozambique" was published in 2019. Journal: BMC Res Notes.

### Discussion

This cost-effectiveness study demonstrates that the new delivery model is the more cost-effective strategy for the universal coverage campaign. The positive incremental net benefit shows that important savings could be achieved from adopting the new delivery model (opportunity-cost).

The ACER per LLIN delivered was lower in the intervention districts. This was mainly driven by the low relative contribution of the micro-planning, LLINs transport, and district-level activities costs. The ACER per HH achieving UC was also lower in the intervention district.

Paintain et al. [12] found higher financial costs for the distribution of LLINs—US$ 1.19 (ranging from US$ 1.08 to US$ 1.41). However, Grabowsky et al. [13] found financial costs of around US$ 0.32, which is considerably lower than what was found in the present study. As for Mueller et al.’s [14], they incurred an ACER of US$ 1.6/LLIN. This ACER is higher than what was found in this study, for either the new or standard delivery model.

From a health-financing point of view, the high overall cost found for these interventions casts doubt on their long-term sustainability in low-income contexts. Mozambique allocated US$ 580.9 million (9% of the National budget) to the health sector in 2015 [15]. For an estimated 25,727,911 inhabitants in 2015 [16], this budget for the health sector corresponds to US$ 22.6 per capita (assuming this as Mozambican State WTP). Taking into account the mean cost to distribute one LLIN with the new intervention (US$ 0.76), and that one LLIN would benefit two persons, the financial sustainability of the intervention would be guaranteed if a campaign were taken stand-alone by the Mozambican State and the WTP were only for the malaria programme (ICER < WTP).

However, considering that the Ministry of Health does not focus exclusively on LLIN campaigns, and other health programmes requires budgetary allocation, the country would not be in a position to guarantee financial sustainability for LLIN distribution. The Mozambique health sector allocated US$ 4,186,129 to the National Malaria Control Programme in 2014 [4]. Considering that 100% of the Mozambican population is at risk for malaria, this allocation corresponds to US$ 0.16 per capita (WTP), i.e., US$ 0.32 for each two persons (US$ 0.44 less than the ACER per LLIN in the intervention). This WTP clearly demonstrates the current financial un-sustainability of the country in assuming the LLINs campaign. The same conclusion holds even considering free warehouse storage, less 50% transport costs, and 50% reduction of LLINs’ purchase cost.

The article "Cost-effectiveness of two long-lasting insecticidal nets delivery models in mass campaign in rural Mozambique" was published in 2019. Journal: BMC Res Notes.

Bed nets campaign is still more cost-effective than indoor residual spraying (US$ 5.41 per person protected) [17], RTS,S (US$ 39.25 per fully vaccinated child) [18, 19], and treatment (US$ 2.59 per person tested and treated) [20]. This is in line with what Winskill et al. [3] found in their modelling cost-effectiveness study. In conclusion, the new delivery model is worthwhile (INB positive) from a programme provider perspective and current donor economic outlook. However, the long-term sustainability of either delivery models is far from guaranteed in Mozambique’s current economic context.

## Limitations

The WTP is often estimated through extensive surveys and is not always available [21]. The rationale for using the three ceiling is not only justifiable, but it is also appropriate to the country context. However, it is suggested that each country should adopt their own value for money ceiling, or make use of net benefit approach with cost-effectiveness acceptability curve if the ceiling is unknown plotting probability of cost-effectiveness against variation of the ceiling. Another limitation is the one-way sensitivity analyses. In the “real-world” more than one parameter varies at a time, and correlation between variation in multiple parameters can overstate uncertainty.

## Data Availability

The datasets used and/or analysed during the current study are available from the corresponding author, upon reasonable request.

## Abbreviations

ACER: average cost-effectiveness ratio
HH/HHs: household/households
ICER: incremental cost-effectiveness ratio
INB: incremental net benefit
LLIN/LLINs: long-lasting insecticidal net/long-lasting insecticidal nets
OR: odds ratio
SA: sensitivity analysis
UC: universal coverage
WTP: willingness-to-pay
